# Clinical Outcomes and Cost Effectiveness of Accelerated Diagnostic Protocol in a Chest Pain Center Compared with Routine Care of Patients with Chest Pain

**DOI:** 10.1371/journal.pone.0117287

**Published:** 2015-01-26

**Authors:** Elad Asher, Haim Reuveni, Nir Shlomo, Yariv Gerber, Roy Beigel, Michael Narodetski, Michael Eldar, Jacob Or, Hanoch Hod, Arie Shamiss, Shlomi Matetzky

**Affiliations:** 1 Leviev Heart Center, Sheba Medical Center, Tel Hashomer, Israel; 2 Ben Gurion University of the Negev, Soroka Medical Center, Beer Sheva, Israel; 3 The School of Public Health, the Sackler Faculty of Medicine, Tel Aviv University, Tel Aviv, Israel; 4 Emergency Medicine Department, Sheba Medical Center, Tel Hashomer, Israel; 5 Sheba Medical Center, Tel Hashomer, Israel; University of Groningen, NETHERLANDS

## Abstract

**Aims:**

The aim of this study was to compare in patients presenting with acute chest pain the clinical outcomes and cost-effectiveness of an accelerated diagnostic protocol utilizing contemporary technology in a chest pain unit versus routine care in an internal medicine department.

**Methods and Results:**

Hospital and 90-day course were prospectively studied in 585 consecutive low-moderate risk acute chest pain patients, of whom 304 were investigated in a designated chest pain center using a pre-specified accelerated diagnostic protocol, while 281 underwent routine care in an internal medicine ward. Hospitalization was longer in the routine care compared with the accelerated diagnostic protocol group (p<0.001). During hospitalization, 298 accelerated diagnostic protocol patients (98%) vs. 57 (20%) routine care patients underwent non-invasive testing, (p<0.001). Throughout the 90-day follow-up, diagnostic imaging testing was performed in 125 (44%) and 26 (9%) patients in the routine care and accelerated diagnostic protocol patients, respectively (p<0.001). Ultimately, most patients in both groups had non-invasive imaging testing. Accelerated diagnostic protocol patients compared with those receiving routine care was associated with a lower incidence of readmissions for chest pain [8 (3%) vs. 24 (9%), p<0.01], and acute coronary syndromes [1 (0.3%) vs. 9 (3.2%), p<0.01], during the follow-up period. The accelerated diagnostic protocol remained a predictor of lower acute coronary syndromes and readmissions after propensity score analysis [OR = 0.28 (CI 95% 0.14–0.59)]. Cost per patient was similar in both groups [($2510 vs. $2703 for the accelerated diagnostic protocol and routine care group, respectively, (p = 0.9)].

**Conclusion:**

An accelerated diagnostic protocol is clinically superior and as cost effective as routine in acute chest pain patients, and may save time and resources.

## Introduction

Chest pain is one of the most common causes of emergency medicine department presentation, accounting for 5–6% of emergency medicine department visits in the United States [1, 2]. The main challenge in evaluating patients with acute chest pain is to identify those with acute coronary syndrome (ACS) where early diagnosis can facilitate effective treatment, while premature discharge may lead to disastrous consequences. In the Unites States, a high 20% of malpractice claims against emergency care physicians relate to management of patients presenting with acute chest pain [3]. The chest pain center concept was developed to address these issues [4–6], and indeed chest pain centers have shown to provide a thorough and fast evaluation by accelerated diagnostic protocol (ADP) for patients presenting with chest pain [7]. Accordingly, in their previously published guidelines, the American Heart Association and the American College of Cardiology implicated the effectiveness of chest pain centers in evaluating patients with acute chest pain [8]. Although experience in the United States has demonstrated that chest pain centers manage patients at low risk for ACS as effectively as in-patient admissions [9–11], current data comprising newer technology, such as coronary multi-detector computed tomography and high sensitive biomarkers, which may facilitate accelerated investigation without compromising its accuracy, are both limited and controversial [12,13]. Moreover, compared with in-patient admissions, the cost effectiveness of chest pain centers and treatment by ADP are debatable [14]. The purpose of this study was to compare cost effectiveness and clinical outcomes of ADP treatment, using newer technology in a specialized chest pain center, with classic routine care for chest pain in a real life setting.

## Methods

### Study design and population

In this comparative prospective study we compared patients with chest pain who were admitted to the Sheba Medical Center (April 2010–August 2011) either to the chest pain center or to one of the internal medicine departments. The Sheba Medical Center is a 1,800 bed tertiary medical center with approximately 192,000 emergency department visits per year, and more than 94,000 admissions annually.

Inclusion criteria included: 1) age ≥18 years; 2) chest pain considered by the attending physician to be suggestive of cardiac origin or requiring admission in order to rule out ACS; 3) absence of baseline electrocardiogram (ECG) changes suggesting acute ischemia or infarction (ST-elevation myocardial infarction, new left bundle branch block, non ST-elevation myocardial infarction or new ST-T changes); 4) absence of elevated cardiac troponin T or I during evaluation in the emergency department; 5) chest x-rays without new pathological findings.

Exclusion criteria included: 1) any reason for chest pain other than ACS that was diagnosed in the emergency department, such as pneumonia, pulmonary embolism, pericarditis or chest trauma; 2) factors such as fever, sepsis, severe anaemia, hyperthyroidism that could exacerbate chronic coronary artery disease; 3) heart failure on admission; 4) unstable angina pectoris, non ST-elevation myocardial infarction or ST-elevation myocardial infarction on admission; 5) any other condition requiring intravenous medication or chronic nursing care; 6) pregnancy.

#### Data collection

Patients were interviewed during their admission course and additional information was collected from patient charts. Three months after discharge, each patient was interviewed by phone. Patients who were found to be eligible and who agreed to participate in the study signed a consent form.

### Study groups

#### The chest pain center group

The center has 8 beds situated in an observation area adjacent to the emergency department. Patients were monitored and observed for a minimum of 8 hours, following which a repeat ECG was performed and cardiac troponin was re-assessed. Each patient was monitored continuously by an ST-segment analyzer. Patients were then referred within the first 24 hours of their admission either to 64-slice multi-detector computed tomography, stress test (exercise ECG), myocardial perfusion study (MPS) with single photon emission computed tomography (SPECT), or stress echocardiography. Discharged patients were followed-up either by a visit to the cardiac outpatient clinic or by a phone call.

#### Internal medicine department (routine care) group

Patients who were suitable candidates for admittance to the chest pain center, but who were eventually admitted to an internal medicine department according to the discretion of the emergency department’s physician. Treatment in the internal medicine department was determined by local internal medicine department protocol for chest pain, at the discretion of the treating physician.

### Data collection and main outcome measures

Data were collected from patient interviews and from their charts, and were followed-up by a phone interview 90 days after discharge.

Independent variables collected included patient history: age, gender, smoking, weight, body mass index; chronic illness (hypertension, diabetes mellitus, dyslipidemia, coronary artery disease; heart failure); previous percutaneous coronary intervention; previous coronary artery bypass graft.

Admission variables included: ECG changes; troponin I, T elevation; percutaneous coronary intervention; coronary artery bypass graft; diagnoses at discharge; recommendations at discharge.

Diagnostic imaging testing during the hospital course included: coronary multi-detector computed tomography; MPS; stress echocardiography.

Dependent variables collected included cardiovascular diagnoses from the chest pain center and internal medicine department and the follow up variables: performing cardiac imaging, coronary revascularization;, readmissions due to recurrent chest pain ACS; death, cardiopulmonary resuscitation; admission and procedure costs, which were calculated using the Israeli Ministry of Health cost list for ambulatory services and admission services 2010 [15].

### Statistical methods

#### Propensity score

Since this was an observational study without random assignment following univariant analysis, inequality was observed in the number of independent variables which could have influenced the outcome variable. Therefore, additional analysis was performed to create a propensity score by using logistic regression. A model of 20 background variables and interactions was designed to calculate predicted probability for all observations to be in the exposure group, i.e. the chest pain center patients. A new continuous variable (0–1) was divided into five strata: from stratum 1 representing low probability to stratum 5 representing high probability of being in the exposure group.

#### Multivariate analysis

Logistic regression was performed to examine differences between the groups in major adverse cardiac events adjusting for propensity score, and results are presented as odds ratio (OR) and confidence interval (CI) of 95%. In addition, Poisson regression was performed to examine differences between the groups for counting outcomes as readmissions and visits to a cardiologist adjusting for propensity score; results are presented as risk ratio (RR) and CI of 95%.

The study was approved by the Sheba Medical Center Institutional Review Board and was supported by the Israel National Institute for Health Policy Research.

## Results

A total of 585 patients were prospectively enrolled (95% response rate). Of them, 304 (52%) were evaluated by ADP in the chest pain center and 281 (48%) were admitted to the internal medicine department and received routine care (Fig. 1). Of the latter, 222 (79%) patients were admitted to the internal ward due to lack of bed availability and 59 (21%) at the discretion of the ED physician.

**Fig 1:** Patients’ enrollment scheme.

### Patient characteristics

Table 1 presents patient characteristics of both study groups. Patients in the routine care group were older and suffered more frequently from hypertension and diabetes mellitus. About one-fourth of the patients in both study groups had sustained prior ACS.

**Table 1:** Patient characteristics

Patient characteristics	RC (N = 281)	ADP (N = 304)	p. value
Age (years) ± SD	60±12	56±11	<0.001
Male gender (%)	182 (65)	201 (66)	0.7
Body mass index ± SD	30±26	28±5.2	0.2
Smokers (%)	80 (29)	94 (31)	0.5
Hypertension (%)	155 (55)	140 (46)	0.03
Diabetes mellitus (%)	97 (35)	59 (19)	<0.001
Dyslipidemia (%)	178 (63)	175 (58)	0.2
Family history of CAD (%)	48 (17)	73 (24)	0.03
Prior ACS (%)	75 (27)	69 (23)	0.3
Prior PCI (%)	89 (32)	68 (22)	0.01
Prior CABG (%)	40 (14)	12 (4)	<0.001
			

RC—Routine care; ADP—Accelerated diagnostic protocol; SD—Standard deviation; CAD—Coronary artery disease; ACS—Acute coronary syndromes; PCI—Percutaneous coronary intervention; CABG—Coronary artery bypass graft.

### Hospital course

Hospitalization stay was longer in the routine care compared with the ADP group (2.61, SD1.07 vs. 2.18, SD 0.98 days, respectively, p<0.001). Nevertheless, the rate of diagnostic imaging testing was significantly higher in the ADP compared with the routine care group [298 (98%) vs. 57 (20%), respectively, p<0.001]. Accordingly, definitive diagnostic workup for rolling out ACS and significant coronary artery disease (CAD) was achieved in significantly higher rates in the ADP group compare with the routine care group [281 (92%) vs. 15 (5%), respectively, p<0.001]. In contrast, the number of blood laboratory tests was significantly higher in the routine care group as shown in Table 2.

**Table 2:** Hospital admission length, procedures and diagnostic imaging testing.

Variables	RC (N = 281)	ADP (N = 304)	p. value
Admission length in days (average ± SD)	2.61±1.07	2.18±0.98	<0.001
SPECT (%)	41 (14)	152 (50)	<0.001
Coronary MDCT (%)	16 (5.7)	139 (45)	<0.001
Stress echocardiography (%)	0 (0)	7 (2.3)	0.02
Coronary angiogram (%)	18 (6.4)	17 (5.6)	0.73
Percutaneous coronary intervention (%)	15 (5.3)	13 (4.3)	0.57
Coronary artery bypass graft (%)	1 (0.4)	2 (0.7)	1.0
Number of CBC tests done (average ± SD)	2.17±0.04	1.12±0.2	<0.005
Number of comprehensive metabolic panel testsdone (average ± SD)	2.25±0.04	2.07±0.03	0.001
Number of CK tests done (average ± SD)	0.83±0.05	0.17±0.03	<0.005
Number of Troponin I tests done (average ± SD)	2.47±0.05	2.18±0.03	<0.005
Number of cholesterol panel tests done(average ± SD)	0.71±0.03	1.01±0.01	<0.005
Recommendation for further ambulatory testing (average ± SD)	124 (44)	13 (4.3)	<0.001

RC—Routine care; ADP—Accelerated diagnostic protocol; SD—Standard deviation; SPECT—single photon emission computed tomography; MDCT—Multi-detector computed tomography; CBC—Complete blood count; CK—Creatine kinase

While in the routine care 244 (87%) patients were discharged with chest pain as the primary diagnosis; 14 (5%) with ACS; 8 (3%) with CAD and 15 (5%) with other diagnoses. In the ADP group, 281 (92%) patients were discharged with non-cardiac chest pain as the primary diagnosis; 9 (3%) with ACS; 9 (3%) with CAD and 5 (2%) with other diagnoses. During the hospital course there were 5 cases of non ST-elevation myocardial infarction in the routine care and none in the ADP patient group (p = 0.025). The discharge recommendations for further ambulatory imaging testing for ruling out significant CAD, were significantly more prevalent in the routine care group [124 (44%) vs. 13 (4.3%), respectively, p<0.001],

### Follow-up results at 3 months

During the 90-day post hospital discharge period, the routine care group of patients were more like to undergo diagnostic imaging tests compared with the ADP patients [125 (44%) vs. 26 (9%), respectively, p<0.001)] (Fig. 2). Ultimately, 70 (25%) patients from the routine care group but only 7 (2%) from the ADP group did not undergo any diagnostic imaging testing within 90 days of index admission (p<0.001). Although cardiac catheterization due to chest pain and/or ACS were more frequent during the follow-up period in the routine care compared with the ADP group [16 (5.7%) vs. 5 (1.6%), respectively, p = 0.01], the number of patients who underwent percutaneous coronary intervention procedures within 90 days of the index hospitalization for chest pain was similar in the two study groups [25 (8.7%) vs. 17 (5.7%), respectively, p = 0.2].

**Fig 2:** Diagnostic imaging testing performed in the community during 90 days of follow-up. RC—Routine care; ADP—Accelerated diagnostic protocol; MPS—Myocardial perfusion scintigraphy; MDCT—Multi-detector computed tomography; Echo—Echocardiography.

Readmissions due to recurrent chest pain during the follow-up period were three times higher in the routine care compared with the ADP group [24 (9%) vs. 8 (3%), p<0.01]. Similarly, routine care patients compared with the ADP group were more likely to sustain ACS (non ST-elevation myocardial infarction or unstable angina pectoris) during the 3-month follow-up period [9 (3.2%) vs. 1 (0.3%), p<0.01] It is important to note that in all ACS events and the vast majority of post discharge readmissions for recurrent chest pain [22 out of 24 (92%)] in the routine care group, occurred among patients who did not undergo complete investigation during the initial hospitalization.

### Multivariate analysis

ADP compared with the routine care was associated with a significant reduction in the ACS rate at 3 months [OR = 0.11 (CI 95% 0.02–0.49)]. This difference remained significant after propensity score analysis [OR = 0.13 (CI 95% 0.03–0.59)]. The ADP group was also associated with a reduction in readmissions due to chest pain within 90 days post discharge compared with the routine care patients [RR = 0.47 (CI 95% 0.31–0.71)], but this difference was only of borderline statistical significant after adjustment for propensity score [RR = 0.68 (CI 95% 0.44–1.07)].

### Cost-effective analysis

The in-hospital costs (admission days, diagnostic tests, blood tests, diagnostic and interventional catheterizations) were similar for the ADP compared with the routine care group [$717,649 ($2,360 per patient) vs. $623,597 ($2,219 per patient), respectively, p = 0.99], as were the post discharge 90-day follow-up costs (re-admissions, diagnostic tests, diagnostic and interventional catheterizations) were higher for the routine care compared with the ADP group [$136,007 ($484 per patient) vs. $45,689 ($150 per patient), respectively, p = 0.74]. Of substantial significance were the ambulatory diagnostic test costs which amounted to $42,877 for the routine care compared with only $8854 for the ADP group. After calculating the overall costs (admission costs plus 90-day follow-up costs), the total cost per patient was $2510 in the ADP compared with $2703 in the routine care group (p = 0.9).

## Discussion

The goal of the present study was to compare the clinical outcome and cost effectiveness of hospitalized patients with chest pain receiving either ADP treatment in a specialized chest pain center or routine care in an internal medicine department in a real-life setting. Overall, the quality of treatment for patients who were evaluated by a pre-determined ADP protocol in a dedicated chest pain center was better with respect to hospitalization length, time from symptom onset to definite diagnosis and, lower readmissions due to chest pain during a 3-month follow-up period, compared with patients treated with routine care. Treatment costs were not higher in the ADP group compared with the patients receiving routine care.

While only 20% of the routine care patients had noninvasive diagnostic imaging testing during the index hospitalization, 98% of ADP patients underwent noninvasive diagnostic imaging with a high rate of coronary multi-detector computed tomography. Accordingly, while 281 (92%) patients in the chest pain center were discharged with a definite diagnosis of non-cardiac chest pain, only 15 (5%) patients who received routine care were discharged with a diagnosis of non-cardiac chest pain. This represents the essence of the ADP approach with its main role of prompt diagnosis and treatment of patients with ACS, and early discharge of patients with non-coronary chest pain [16, 17].

Recent studies have showed that the use of coronary multi-detector computed tomography and high sensitive biomarkers, which play a pivotal role in the ADP, facilitate accelerated investigation without compromising its accuracy. It facilitates rapid evaluation, requires minimal patient cooperation (short breath hold), is fast and has high diagnostic accuracy [12–13, 18]. The ROMICAT-I and other studies [18–20] have shown that normal findings on multi-detector computed tomography have a very high negative predicting value for ruling out ACS during the index hospitalization and for the occurrence of major adverse cardiac events over the following two years. Therefore, it is safe to discharge chest pain center patients, even after a very short hospitalization stay, with high assurance that they will do well with very low major adverse cardiac events. Moreover, the use of high sensitive troponin facilitates even further the discharge of the chest pain center patients after a relatively short hospitalization course [21, 22]. On the other hand the heavy work load in the internal medicine department might have compromised the capability of accurately diagnosing many patients with chest pain, by avoiding necessary noninvasive stress tests, and by spending precious time carrying out unnecessary tests [23–25]. The uncertainty regarding diagnosis and the need for further completion of diagnostic testing, could cause anxiety, defensive medicine [26, 27] and explain the high rates of readmission [28, 29]. On the other hand patients who were “already worked up” in the chest pain unit and had a negative coronary CT would not be re-admitted even when they came back with chest pain. Indeed, most of the readmissions for ACS occurred in the routine care arm in patients who did not undergo complete evaluation during the initial hospitalization. Furthermore, although the rate of coronary revascularization did not differ between the two study groups, patients in the ADP as compared to the routine care group underwent the revascularization procedure much earlier, during the initial hospitalization.

Finally, the ADP treatment costs were not higher than the routine care costs, even when cost analysis for loss of workdays for patients who had to complete their diagnostic tests in the community were not included, a fact which could cause routine care costs to be even higher [17, 30–31]. Furthermore, for cost analysis purposes, we calculated the length of stay by days and not hours, but in actual fact no patient stayed for longer than 24 hours in the chest pain center.

### Study Limitations

The study was a single-center study; nevertheless, it was carried out in a large tertiary medical center.

The study was not randomized and hence patient baseline characteristics were different. Accordingly the reason for increased rate of ACS in the routine care group of patients may be the higher risk characteristics of patients in this arm.

## Conclusions

Although the non randomized design of the study is an important limitation, we believe that our findings suggest that fast and definitive investigation of patients with acute chest pain according to pre-specified protocol provides better quality of care with shorten hospitalization length, time to definite diagnosis and, lower readmissions rate compared with patients treated with routine care and might even reduce healthcare expenses This approach can also contribute towards lowering the workload and burden in the internal medicine department. Yet, further larger randomized studies are needed to support these findings.
